The article "In-vitro and in-vivo validation of ethnopharmacological uses of methanol extract of Isodon rugosus Wall. ex Benth. (Lamiaceae)" was published in 2014. Journal: BMC Complement Altern Med.

# *In-vitro* and *in-vivo* validation of ethnopharmacological uses of methanol extract of *Isodon rugosus* Wall. ex Benth. (*Lamiaceae*)

**DOI:** 10.1186/1472-6882-14-71

**Published:** 2014-02-22

**Authors:** Khalid Hussain Janbaz, Javeria Arif, Fatima Saqib, Imran Imran, Muhammad Ashraf, Muhammad Zia-Ul-Haq, Hawa ZE Jaafar, Vincenzo De Feo

**Affiliations:** 1 Faculty of Pharmacy, Bahauddin Zakariya University, Multan, Pakistan; 2 Department of Biochemistry and Biotechnology, Islamia University, Bahawalpur, Pakistan; 3 The Patent Office, Karachi, Pakistan; 4 Department of Crop Science, Faculty of Agriculture, 43400 UPM Serdang, Selangor, Pakistan; 5 Department of Pharmacy, Salerno University, Fisciano, Salerno, Pakistan

**Keywords:** *Isodon rugosus*, Traditional uses, Spasmogenic activity, Spasmolytic activity, Analgesic activity

## Abstract

**Background:**

*Isodon rugosus* is used in folk Pakistan traditional practices to cure ailments related to gastrointestinal, respiratory and cardiovascular problems. Present study was undertaken to validate these folkloric uses.

**Methods:**

A crude methanol extract of the aerial parts of *Isodon rugosus* (Ir.Cr.) was used for both *in vitro and in vivo* experiments. The plant extract was tested on isolated rabbit jejunum preparations for possible presence of spasmolytic activity. Moreover, isolated rabbit tracheal and aorta preparations were used to ascertain the relaxant effects of the extract. Acetylcholinesterase and butyrylcholinesterase inhibitory activities of Ir.Cr were also determined as well as its antioxidant activity. The *in vivo* antiemetic activity of the extract was evaluated by using the chick emesis model, while the analgesic and antipyretic activities were conducted on albino mice.

**Results:**

The application of the crude extract of *I. rugosus* to isolated rabbit jejunum preparations exhibited relaxant effect (0.01-0.3 mg/ml). The Ir.Cr also relaxed K^+^(80 m M)-induced spastic contractions in isolated rabbit jejunum preparations and shifted the Ca^+2^ concentration response curves towards right (0.01-0.3 mg/ml). Similarly, the extract, when applied to the isolated rabbit tracheal preparations relaxed the carbachol (1 M)- as well as K^+^ (80 mM)-induced contractions in a concentration range of 0.01-1.0 mg/ml. Moreover, it also relaxed (0.01-3.0 mg/ml) the phenylephrine (1 M)- and K^+^ (80 mM)-induced contractions in isolated rabbit aorta preparations. The Ir.Cr (80 mg/kg) demonstrated antipyretic activity on pyrogen-induced pyrexia in rabbits as compared to aspirin as standard drug. The Ir.Cr also exhibited anti-oxidant as well as inhibitory effect on acetyl- and butyryl- cholinesterase and lipoxygenase (0.5 mg/ml).

**Conclusions:**

The observed relaxant effect on isolated rabbit jejunum, trachea and aorta preparations caused by Ir.Cr is possibly to be mediated through Ca^+2^ channel blockade and therefore may provided scientific basis to validate the folkloric uses of the plant in the management of gastrointestinal, respiratory and cardiovascular ailments. The observed antioxidant activity as well as the lipoxygenase inhibitory activity may validate its traditional use in pain and inflammations.

## Background

*Isodon rugosus* Wall. ex Benth. (*Lamiaceae*), locally known as boi, sperkai and phaypush, is found in Northern areas of Pakistan [1-4]. The plant is an aromatic, branched shrub, 1-5 ft in height, with erect stem, ovate leaves of notched margin and covered with dense small hairs on ventral side. It flowers from July to September and the seeds ripen from August to October [5].

The plant is used in traditional medical practices in tooth ache and is claimed to be effective as an antiseptic, a hypoglycaemic, an anti-diarrheal and a bronchodilator [2,3]. A topical administration of fresh leaf extract is used to treat scabies for its immediate effect, while 1-2 drops of this extract are used to treat earache [6]. An extract of leaves is also used to treat hypertension, fevers, rheumatism and toothache. Branches are used for making dusters [1,7].

Previous phytochemical investigation of the plant revealed the presence of steroids, flavonoids, terpenoids, saponin, tannins, cardiac glycosides, coumarins, reducing sugars and β-cyanin among the methanol soluble extractable constituents. From the plant, some diterpenoids, *i.e.* rugosinin, effusanin-A, effusanin-B, effusanin-E, lasiokaurin and oridonin, have been isolated. The compounds exhibited DNA protective activity in yeast strains [8,9]. Moreover, the analysis of volatile oil fractions from leaves and inflorescence indicated presence of sesquiterpene hydrocarbons, including β-caryophyllene, germacrene-D and α-humulene as the major constituents [10]. Furthermore, plant extracts and fractions by different solvents exhibited antifungal [5], antibacterial, phytotoxic [11] and antioxidant activities [12].

Smooth muscle contractile activity plays a vital role in regulating functions of gastrointestinal (GIT), respiratory and cardiovascular systems in human body. Malfunction of smooth muscle contractility in any of these systems leads to many GIT disorders like intestinal spasms and cramps; cardiovascular disorders like hypertension and hypotension and airway disorders like asthma. Smooth muscle activity is regulated by the cytosolic Ca^2+^ level, and the sensitivity to Ca^2+^ of the contractile elements in response to changes in the environment surrounding the cell [13]. Plant extracts can stimulate, coordinate, and restore smooth muscle activity of gastrointestinal (GIT), respiratory and cardiovascular systems. Since rabbit GIT, aorta as well as trachea shares many physiological, anatomical and pharmacological similarities of similar human organs and are therefore used to study effect plant on smooth muscle. There are many studies describing effect of plant extracts on isolated smooth muscle tissue of various animal models including rabbit [14-29]. Natural analgesics are used to control pain. Analgesic activity of plant extracts is evaluated using various animal models, the most common being tail flick model due to its reliability and minimal interanimal variation. Many studies have been carried out by using this model [30-34]. Similarly chick emesis model is mostly used in Pakistan [35-39].

Despite the tagged multiple therapeutic benefits of *I. Rugosus* in asthma, GIT, cardiovascular problems as well as its use as anti-emetic and analgesic remedy, no data is available with respect to its effectiveness in ailments of any of these vital organs of human body. The present study on the crude extract of *I. rugosus* and its fractions was undertaken using various pharmacological models to rationalize these traditional uses and to explore mechanistic basis for these medicinal uses.

## Methods

### Collection of Plant and preparation of extract

The aerial parts of *Isodon* rugosus were collected from the rural areas of Swat, Pakistan in September, 2011. The plant was identified by the taxonomist, Ms Saima Shehzadi from the Institute of Pure and Applied Biology, Bahauddin Zakariya University, Multan and a voucher specimen of the plant was deposited in the herbarium of this Institute (voucher # F.P.241-5). The plant material was shade dried, rendered free of adulterants and grinded into coarse powder*.* Approximately 500 g powdered plant material was soaked in 80% aqueous-methanol by cold maceration at room temperature for 7 days with occasional shaking. The filtration through Whatman-1 filter paper was preceded by passage through a muslin cloth to avoid choking by vegetative debris. The filtrate was evaporated to a brownish green extract under reduced pressure on a rotary evaporator at room temperature, with a yield of 12%. The stock solutions of *Isodon* rugosus were prepared in distilled water and the dilutions were made fresh in normal saline on the day of experiment.

### Chemicals

Acetylcholine chloride, atropine sulfate, carbachol, histamine, isoprenaline, pyrillamine, potassium chloride, verapamil hydrochloride and phenylephrine, magnesium chloride, ethylene tetra-acetic acid (EDTA) were purchased from Sigma Chemicals Co. St. Louis, MO, USA. Calcium chloride, glucose, magnesium sulphate, potassium dihydrogen phosphate, sodium bicarbonate, sodium dihydrogen phosphate, and methanol were obtained from Merck, Darmstadt, Germany. Ammonium hydroxide, sodium chloride, and sodium hydroxide were purchased from BDH Laboratory supplies, Poole, England. The above-mentioned chemicals were of highest purity and reagent analytical research grade.

### Animals and housing conditions

Animals (♂/♀) used in this study were local strain rabbits (1.0-1.8 kg), mice (Swiss albino 28-30 g) and chicks (white leghorn meant for laying eggs). Animals were housed under controlled environmental condition (23-25°C) at the animal house of Faculty of Pharmacy, Bahauddin Zakariya University, Multan. The animals were provided with standard food and tap water *ad libitum.* The animals were deprived of food 24 hr prior to the experiments but were given free access to water. Rabbits were sacrificed following a blow on back of head to be used for *in vitro* studies. All the experiments performed complied with the rulings of Institute of Laboratory Animal Resources, Commission on Life Sciences [40]. The experimental protocols regarding current study were submitted to and approved by the ethical committee meeting held on 14-02-2011 via Notification Number EC/02/2011 dated of the Department of Pharmacy, Bahauddin Zakariya University, Multan.

### Experiments on isolated tissues

The experiments on isolated tissues were performed by adoption of procedures as described previously [24-27]. Briefly, we used freshly prepared jejunum, tracheal and aortic tissue segments from the rabbit and maintained adequately in the respective buffer solutions. The detailed elaboration of each tissue extraction procedure is described below under the respective heading (a-c).

#### ***Isolated rabbit jejunum preparations***

The plant extract was tested on isolated rabbit jejunum preparations for detecting a possible presence of spasmolytic activity. Rabbit was dissected to remove jejunum and this was placed in a Tyrode physiological salt solution maintained at 37°C and aerated with carbogen (95% O_2_ and 5% CO_2_). The tissue were cut into segments of about 2 cm in length, rendered free of adhering mesenteries and were subsequently suspended in isolated tissue baths containing Tyrode’s solution, at 37°C and aerated with carbogen. The composition of the Tyrode’s solution (mM) was: KCl (2.68), NaCl (136.9), MgCl_2_ (1.05), NaHCO_3_ (11.90), NaH_2_PO_4_ (0.42), CaCl_2_ (1.8) and glucose (5.55). A preload tension of 1 g was applied and intestinal contractions were recorded isotonically through a Powerlab Data Acquisition System (AD Instruments, Sydney, Australia). The tissues were allowed to equilibrate for about 30 min prior to exposure to any test material. The isolated rabbit jejunum preparations exhibit spontaneous rhythmic contractions and allow testing of the relaxant (spasmolytic) effect without application of an agonist [25]. The response observed on addition of test material to isolated tissue bath was quantified by dose addition in cumulative manner. The observed relaxant effects of test substance were quantified as the percent decrease in spontaneous contractions of the preparation recorded immediately prior to the addition of test substances. The possible mechanism of the relaxant activity of the test material was investigated through the relaxation of K^+^ (80 mM)-induced sustained spasmodic contractions [25,27]. The test material was added to isolated tissue bath in a cumulative manner to relax sustained contractions in concentration-dependent manner. The observed relaxant effect of the test material on K^+^ (80 mM)- induced contraction was expressed as percent of the control contractile response.

Calcium channel blocking effect of the test substance was confirmed by the method described previously [24,26]. The isolated rabbit jejunum preparation was allowed to stabilize in normal Tyrode’s solution, which was subsequently replaced for 30 min with Ca^2+^-free Tyrode’s solution to which EDTA (0.1 mM) was added in order to remove calcium from the tissue. The isolated tissue bath solution was further replaced with K^+^-rich and Ca^2+^- free Tyrode’ssolution, having the following composition (mM): KCl (50), NaCl (91.04), MgCl_2_ (1.05), NaHCO_3_ (11.90), NaH_2_PO_4_ (0.42), glucose (5.55) and EDTA (0.1). Subsequent to an incubation period of 30 min, Ca^2+^ was added to the tissue bath in cumulative manner to obtain control calcium concentration response curves (CRCs). The CRCs were prepared in duplicate and tissue was then washed and allowed to be equilibrated in the presence of plant extract for 1 hour prior to recording of the concentration response curves of Ca^2+^ for comparison to the control concentration response curves. The CRCs of Ca^2+^ were recorded in the presence of different concentrations of the plant extract in tissue bath.

#### ***Isolated rabbit tracheal preparations***

Rabbit trachea was dissected out as described previously [27,41] and kept in a Krebs solution having the following composition (mM): NaCl (118.2), NaHCO_3_ (25.0), CaCl_2_ (2.5), KCl (4.7), KH_2_PO_4_ (1.3), MgSO_4_ (1.2) and glucose (11.7). The trachea was cleaned free from the surrounding fatty tissues and rings of 2–3 mm width containing 2–3 cartilages were prepared. Each ring was opened by a longitudinal incision on the ventral side opposite to the smooth muscles layer to form a strip with smooth muscles layer in middle and cartilages on both sides. These tracheal tissues were mounted in 20 ml organ bath containing the Krebs solution being maintained at 37°C and aerated with carbogen. A preload tension of 1 g was applied and tissue preparations were allowed to be equilibrated for 1 hour prior to any challenge by the drug. The Ir.Cr was added to the isolated tissue bath in different concentrations in cumulative manner to assess the possible relaxant effect on carbachol (1 μM)- and high K + (80 mM)-induced sustained contractions. The isometric contractile responses were recorded through a Powerlab Data Acquisition System (AD Instruments, Sydney, Australia) linked to a computer installed with a Lab Chart software (Version 7). The standard drug, Verapamil, with Ca^2+^ channel blocking effect, was tested on carbachol (1 μM)- and K^+^ (80 mM)- induced spastic contractions to evaluate the possible mode of action.

#### ***Isolated rabbit aorta preparation***

The descending thoracic aorta was dissected out and kept in Krebs solution at 37°C and aerated with carbogen. It was cut into rings of about 2–3 mm in width and each ring and was mounted in a tissue bath containing the Krebs solution at 37°C and aerated with carbogen. A preload tension of 2 g was applied to each preparation and allowed to equilibrate for a period of 1 hour. Vasorelaxant effects of Ir.Cr were assessed on phenylephrine (1 μM)- and K^+^ (80 mM)-induced spastic contractions in isolated tissue preparations. Changes in isometric tension of aortic rings were recorded via a force-displacement transducer coupled to a Powerlab Data Acquisition System (AD Instruments, Sydney, Australia) linked to a computer installed with Lab Chart software (version 7).

### Cholinesterases and lipoxygenase activity

The acetylcholinesterase (AChE electrical eel, Type VI-S, EC 3.1.1.7; Sigma) and butyrylcholinesterase (BuChE equine serum EC 3.1.1.8; Sigma) inhibitory activities of Ir.Cr were determined subsequent to minor modification of previously reported spectrophotometric method [42] by using 96-well plate reader Synergy HT, Biotek, USA, taking eserine (0.25 mM per well) as standard inhibitor. The acetylcholinesterase/butyrylcholinesterase activity was estimated following hydrolysis of substrate like acetylthiocholine/butyrylthiocholine (Sigma) by respective cholinesterases into thiocholine, which on reaction with 5,5′-dithiobis(2-nitrobenzoic acid) (DTNB) produced a yellow product (5-thio-2-nitrobenzoic acid) at PH 8 and maximum absorbance was measured at 405 nm after 15 min incubation at 37°C. The inhibitory influence of Ir.Cr (0.5 mg/ml) and eserine (0.25 mM) on AChE and BuChE activity was assessed by repeating the above-mentioned procedure in the presence of test compounds in the reaction mixture. Ethanol was taken as negative control. The IC_50_ values were determined on addition of multiple dilution of Ir.Cr (i.e. 0.5, 0.25, 0.125, 0.0625, 0.0313, 0.015 mg/ml) and eserine (i.e. 0.5, 0.25, 0.125, 0.0625, 0.0313, 0.015 mM) to the reaction mixtures and data obtained was analyzed on EZ–Fit Enzyme kinetics software (Perrella Scientific Inc. Amherst, USA) decrease in absorbance indicated increase in enzyme inhibitory activity. Moreover, the lipoxygenase (LOX) inhibitory activity was assayed following the method proposed by Tappel [43].

The decrease in absorbance indicates increased enzyme inhibition activity which was determined by the following formula.

$$\begin{array}{ll} \text{Inhibition}\left(\%\right)= & \left(\text{Abs}.\mathrm{of}\;\text{control}–\text{Abs}.\mathrm{of}\;\text{test}\;\text{solution}\right)\\ & \times 100\;\mathrm{Abs}.\mathrm{of}\;\text{control} \end{array}$$

Where

$$\begin{array}{ll} \text{Absorbance}\;\mathrm{of}\;\text{Control}= & \text{Total}\;\text{enzyme}\;\text{activity}\\ & \text{without}\;\text{inhibitor} \end{array}$$

$$\begin{array}{ll} \text{Absorbance}\;\mathrm{of}\;\text{Test}= & \text{Activity}\;\mathrm{in}\;\text{the}\;\text{presence}\;\mathrm{of}\\ & \text{test}\;\text{compound} \end{array}$$

### Determination of antioxidant activity

The antioxidant activity was determined by DPPH assay, which was carried out following the protocol of previously reported method [44]. Ascorbic acid was used as a standard antioxidant and all experiments were carried out in triplicates. The reduction in the absorbance was measured at 517 nm using a Synergy HT BioTek^®^ USA microplate reader and data obtained was computed on Ez-fit software.

### Anti-emetic activity

The antiemetic activity of the Ir.Cr was evaluated by using chick emesis model [45]. The chicks were placed under large beakers and were acclimatized for 30 min. The animals of group 1 (n = 5) were given an oral dose of normal saline and copper sulphate was given orally (50 mg/kg) about 10 min after the last treatment. The group 2 animals (n = 5) were treated similar to group 1 except normal saline was replaced by Ir.Cr (150 mg/kg; solubilised in normal saline). Whereas, the group 3 of animals (n = 5) were treated similar to group 2 of animals except chlorpromazine (150 mg/kg) was substituted for Ir.Cr. The numbers of retches were counted during the next 10 minutes and the percent inhibition was evaluated by the formula as given below:

$$“\text{Inhibition}\left(\%\right)=\left(A-B/A\right)x100”$$

Where,

A=Frequencyofretchingincontrolgroup

B=Frequencyofretchingintestgroup

### Analgesic activity

The screening for analgesic activity was conducted on albino mice subsequent to minor modifications of the previously reported technique [46]. The tails of mice were dipped in water maintained at 55°C, while holding animals in vertical position. The time taken by mice to withdraw its tail out of water was the reaction time. The reaction time was noted prior to treatment of a group of mice (n = 5) and Ir.Cr (200 mg/kg; i.p., dissolved in normal saline) was injected after 10 min of noting reaction time and reaction time was noted after 15 min of Ir.Cr treatment. In a similar group of mice (n = 5), the above-mentioned procedure was repeated except aspirin (75 mg/kg; I.P) was substituted for Ir.Cr.

### Antipyretic activity

The Ir.Cr was subjected to screening for possible antipyretic activity following minor modification of the previously reported method [47]. The albino rabbits (1-1.5 kg) were divided in to 3 groups each containing 5 animals. The group 1 animals were regarded as control, and was given an i.p. injection (0.5 ml/kg) of pyrogen (brewer yeast) and an injection of normal saline (2 ml/kg) about 40 min of after first treatment. The group 2 animals were designated as experimental and were treated similar to group 1 animals except the Ir.Cr (80 mg/kg) dissolved in normal saline (2 ml) was substituted for normal saline. The group 3 animals were considered as standard and received treatment similar to group 2 animals except aspirin (10 mg/kg) dissolved in normal saline (2 ml) was injected intraperitoneally. The rectal temperatures of the rabbits were noted after every 5 min with clinical thermometer by inserting to the rectum to the extent of about 0.5 cm subsequent to lubrication of thermometer bulb with glycerine till the temperature become normal.

### Statistical analysis

The values were expressed as mean ± standard error (Mean ± SE). Student’s t-test was applied for assessment of observations. P < 0.05 was believed to be statistically significant.

## Results

### Effect of Ir.Cr on isolated rabbit jejunum preparations

The application of the methanol extract of *Isodon rugosus* to the isolated rabbit jejunum preparations exerted relaxant effect at a tissue bath concentration range of 0.1-0.3 mg/ml, with an EC_50_ value of 0.16 mg/ml (95% CI:0.01-0.291; n = 5) (Figure 1). The Ir.Cr also caused relaxation of K^+^(80 mM)-induced spastic contractions at a tissue bath concentration of 0.3 mg/ml and EC_50_ value of 0.15 mg/ml (95% CI:0.01-0.29; n = 5) (Figure 2). The Ir.Cr-induced relaxant effect was found to be comparable to the effect of the standard drug, verapamil, which relaxed the spontaneous and K^+^(80 mM)-induced contractions with respective EC_50_ value of 0.65 μM (95%CI:0.5551-0.8601; n = 5) and 0.70 μM (95% CI:0.5777-0.8881; n = 5) (Figure 2).

**Figure 1:** **Tracings showing (a) spontaneous contraction of isolated rabbit jejunum and (b) spasmolytic effect of the crude extract of *Isodon rugosus *(Ir.Cr).** Plant extract was added in cumulative manner and values listed were the final tissue bath concentrations, (n = 5).

**Figure 2:** **Concentration dependent relaxant effect of (a and b) methanol extract of *Isodon rugosus *(Ir.Cr) and (c) verapamil on spontaneous and high K + (80 mM)- induced contractions in isolated rabbit jejunum preparations.** Values are the mean ± SEM, n = 5.

To assess the potential Ca^2+^ antagonistic effect, Ir.Cr was also tested on the control concentration response curve of calcium. The medium was Ca^2+^ free and the spontaneous contractions of the isolated rabbit jejunum preparations were eradicated completely but the cumulative addition of Ca^2+^ (0.1–6.4 mM) caused a stepwise restoration of the contractile activity in tissue and maximal contraction was attained at tissue bath concentration of 6.4 mM of Ca^2+^, which was assumed to be 100%. Subsequently, the jejunum tissue incubated with Ir.Cr at a concentration range of 0.1–0.3 mg/ml for 35 min shifted the concentration response curve of Ca^2+^ towards right. These effects were found to be similar to those produced by verapamil (0.1–0.5 μM), (Figure 3, n = 5).

**Figure 3:** **Effect of (a) methanol extract of *Isodon rugosus *(Ir.Cr) and (b) verapamil on concentration response curves of Ca**^**2+ **^**in isolated rabbit jejunum preparations.** Values are the mean ± SEM, n = 5.

### Effect of Ir.Cr on isolated rabbit tracheal preparations

The Ir.Cr caused relaxation of the carbachol (CCh) (1 μM)- and K^+^ (80 mM)–induced contractions in isolated rabbit tracheal preparations at the tissue bath concentrations ranging from 0.1 to 0.3 mg/ml, with respective EC_50_ value of 0.22 mg/ml (95% CI:0.01-0.74; n = 5) and 0.20 mg/ml (95% CI:0.01-0.57; n = 5) (Figure 4a,b,c). Similarly, verapamil relaxed the CCh (1 μM)- induced contractions with EC_50_ of 0.6910 mg/ml (95% CI:0.5551-0.8601; n = 5), as well as K^+^(80 mM)-induced contractions with EC_50_ of 0.6910 mg/ml (95% CI:0.5551-0.8601; n = 5) (Figure 4d).

**Figure 4:** **Concentration dependent inhibitory effect of (a, b and c) methanolic extract of *Isodon rugosus *(Ir.Cr) and (d) verapamil on carbachol (1 μM)- and high K**^**+ **^**(80 mM)- induced contractions in isolated rabbit tracheal preparations.** Values are the mean ± SEM, n = 5.

### Effect of Ir.Cr on isolated rabbit aorta preparations

The Ir.Cr exhibited relaxant effect on isolated rabbit aorta preparations. It caused relaxation of K^+^ (80 mM) and phenylephrine (1 μM)-induced contractions with EC_50_ values of 0.21 mg/ml (95% CI:0.011-0.57; n = 5) and 1.43 mg/ml (95% CI:0.01-2.74; n = 5), respectively (Figure 5a,b,c). These effects were comparable to those of verapamil, which relaxed the phenylephrine- and K^+^(80 mM)- induced contractions with respective EC_50_ of 0.90 μM (95% CI:0.03-5.02; n = 5) and 0.43 μM (95% CI: 0.03-1.98; n = 5) (Figure 5d).

**Figure 5:** **Concentration dependant inhibitory effect of (a, b and c) methanolic extract of *Isodon rugosus *(Ir.Cr) and (d) verapamil on phenylephrine (1 μM)- and high K + (80 mM)- induced contractions in isolated rabbit aorta preparations.** Values are the mean ± SEM, n = 5.

### Effect of Ir.Cr on cholinesaterases and lipoxygenase enzymatic activity

The methanol extract of *Isodon rugosus* caused 41.66 ± 0.3% inhibition of AChE activity at a concentration of 0.5 mg/ml, while the standard drug, eserine, caused an inhibition of 91.29 ± 1.17% of AChE activity at 0.25 mM concentration. The IC_50_ value for AChE after Ir.Cr administration was 0.6 ± 0.04 mg/ml, whereas for eserine it was estimated as 0.14 ± 0.001 mM (Table 1).

**Table 1:** Inhibitory activity of Ir.Cr on cholinesterases and lipoxygenase enzymatic activities in comparison to respective standards

**Enzymatic activity**	**Test material**	**Conc./well**	**% Inhibition**	**IC**_**50**_
Acetylcholinesterase	Ir.Cr	0.5 mg/ml	41.66 ± 0.3	0.6 ± 0.04 mg/ml
	Eserine*	0.25 mM	91.29 ± 1.17	0.14 ± 0.001 mM
Butyrylcholinesaterase	Ir.Cr	0.5 mg/ml	33.78 ± 0.5	0.74 ± 0.02 mg/ml
	Eserine	0.25 mM	82.82 ± 1.09	0.15 ± 0.02 mM
Lipoxygenase	Ir.Cr	0.5 mg/ml	36.65 ± 2.8	0.68 ± 0.07 mg/ml
	Baicalin**	0.25 mM	93.79 ± 1.38	0.13 ± 0.015 mM

*Standard for cholinesterases; **standard for lipoxygenase.

The Ir.Cr caused 33.78 ± 0.5% inhibition of butyrylcholinesterase (BchE) enzyme at a concentration of 0.5 mg/ml, whereas eserine exhibited 82.82 ± 1.09 inhibition of BchE at 0.25 mM concentration. The IC_50_ value of Ir.Cr for BchE was found to be 0.74 ± 0.02 mg/ml, whereas it was calculated to be 0.15 ± 0.02 μM for serine (Table 1).

The extract (0.5 mg/ml) exerted 36.65 ± 2.8% inhibition of lipoxygenase in comparison to the standard durg, baicalin (0.25 mM/L), which exhibited 93.79 ± 1.38% inhibition. The IC_50_ for Ir.Cr and baicalin was 0.68 ± 0.07 mg/ml and 0.13 ± 0.015 mM, respectively (Table 1).

### Anti-oxidant activity of Ir.Cr

The Ir.Cr exhibited 41.26 ± 0.2% scavenging activity against DPPH at a concentration of 0.5 mg/ml as compared to the standard ascorbic acid, which showed 92 ± 0.1% activity (Table 2).

**Table 2:** Anti-oxidant activity of Ir.Cr

**Sample**	**Concentration**	**% Inhibition**
Ir.Cr	0.5 mg/ml	41.26 ± 0.02
Ascorbic acid	0.3 mM/L	92 ± 0.1

### Anti-emetic activity of Ir.Cr

In the control group of animals to whom normal saline (10 ml/kg) followed by the emetic copper sulphate (50 mg/kg) was administered orally, the number of retches were 58.8 ± 0.1. The group of animals was treated similarly, but Ir.Cr (150 mg/kg) substituted the normal saline, showed a significantly reduced number of retches (46.2 ± 0.3) (p <0.01). This value was found to be comparable to a group of animals treated with the standard anti-emetic, chlorpromazine (150 mg/kg), where retches were significantly (p <0.01) decreased to 46.0 ± 0.2. Thus Ir.Cr (150 mg/kg) exhibited a significant antiemetic activity (21.42%; p < 0.01), in a manner comparable to chlorpromazine (150 mg/kg) as standard drug (21.76%; p < 0.01) (Table 3).

**Table 3:** Anti-emetic effect of Ir.Cr in comparison to chlorpromazine

**Groups**	**No. of retches ± S.E.M**	**% Inhibition of emesis**
Control (10 ml/kg)	58.8 ± 0.1	Nil
Chlorpromazine (150 mg/kg)	46.0 ± 0.2	21.76
Ir.Cr (150/mg/kg)	46.2 ± 0.3	21.42

### Analgesic activity of Ir.Cr

The duration of tail deflection prior to drug administration was 2.73 ± 0.01 s, but Ir.Cr (200 mg/kg; i.p., diluted in saline) treatment resulted in a significantly (p <0.01) increased deflection time, i.e., 9.35 ± 0.08 s. Similarly, the treatment with aspirin (75 mg/kg; i.p. diluted in saline) also resulted in a significant (p <0.01) increase in tail deflection time in mice (9.62 ± 0.2 s). Thus, Ir.Cr treatment exerted analgesic effect in mice in terms of increase in tail deflection time in a manner similar to aspirin used as a standard analgesic drug (Table 4).

**Table 4:** Effect of Ir.Cr and aspirin on tail deflection time (s) in mice

**Groups**	**Control**	**Treated**	**Standard**
**Dosage**	**Saline 10 ml/kg**	**Ir.Cr 200 mg/kg**	**Aspirin 75 mg/kg**
**Tail deflection time (seconds)**	2.73 ± 0.1	9.35 ± 0.8	9.62 ± 0.2

### Antipyretic effect of Ir.Cr

Animals of control group, to whom (0.5 ml/kg; i.p.) of pyrogen (brewer yeast) was injected at 0 time, presented a rectal temperature of 38.44 ± 0.1°C. Two hrs after normal saline was injected subsequent and rectal temperature was 40.16 ± 0.2°C. The values of rectal temperature at 3, 4 and 5 hrs were 40.12 ± 0.1, 40.10 ± 0.01 and 40.10 ± 0.1°C, respectively. The animals of treated group received a similar treatment except for administration of Ir.Cr (80 mg/kg; i.p., diluted in saline) in substitution of saline; the rectal temperatures at 0, 2, 3, 4 and 5 hrs 37.9 ± 0.2, 39.05 ± 0.05, 38.85 ± 0.07, 38.38 ± 0.2, and 38.38 ± 0.1°C, respectively. The animals of aspirin group received a similar treatment except for administration of aspirin (10 mg/kg; i.p., diluted in saline) and temperatures noted at 0, 2, 3, 4 and 5 hrs were 38.93 ± 0.1, 38.71 ± 0.2, 38.06 ± 0.1, 38.32 ± 0.2, and 39.20 ± 0.1°C, respectively. There was a significant (P < 0.05) rise in temperature subsequent to pyrogen injection in all the control group of animals but only Ir.Cr and aspirin treatments resulted in significant decrease in body temperature, thus indicating a potential antipyretic effect of Ir.Cr (Table 5).

**Table 5:** Effect of Ir.Cr on pyrogen-induced pyrexia in rabbit

**Groups**	**Treatment**	**Rectal temperatures**				
		**0 hr**	**2 hs**	**3 hs**	**4 hs**	**5 hs**
Control	Pyrogen + Saline	38.44 ± 0.1	40.16 ± 0.2	40.12 ± 0.1	40.10 ± 0.1	40.10 ± 0.1
Ir.Cr	Pyrogen + Ir.Cr 80 mg/kg	37.9 ± 0.2	39.05 ± 0.05	38.85 ± 0.07	38.37 ± 0.02	38.37 ± 0.03
Aspirin	Pyrogen + Aspirin 10 mg/kg	38.93 ± 0.1	38.71 ± 0.2	38.06 ± 0.1	38.32 ± 0.2	39.20 ± 0.1

## Discussion

*Isodon rugosus* has folkloric repute to be beneficial in the management of multiple ailments pertaining to gastrointestinal, respiratory and cardiovascular systems. GIT disorders such as, indigestion and constipation are believed as root cause of many diseases and indigenous communities in Pakistan use plant parts to cure them as herbal therapy. The present study was undertaken for the scientific validation of these folkloric claims through an exploration of the possible mechanism(s) of action.

The application of the methanol extract of *Isodon rugosus* to the spontaneously contracting isolated rabbit jejunum preparations showed a relaxant effect, as reflected by decrease in both amplitude and frequency of the spontaneous contractions. The spontaneous movements of intestine is a phenomenon of alternative depolarization and repolarization and the maximal depolarization is mediated through action potential produced via rapid influx of Ca^2+^ by means of voltage dependant L-type Ca^2+^ channels (VDLCs) [48]. The increased availability of Ca^2+^ in cytoplasm results in enhanced contraction of smooth muscle preparations through activation of several nero-endocrinal agonists, i.e., acetylcholine, histamine and serotonin [49].

The possible mechanism of observed relaxant effect by the extract was tested against the K^+^(80 mM)-induced contractions in isolated rabbit jejunum. The exposure to K^+^(>30 mM) can induce contraction of smooth muscles through opening of voltage dependent calcium channels, increased influx of extracellular Ca^+2^ leading to contractile effect [50]. The substances capable to relax K^+^ (80 mM)-induced contractions are speculated to act through blockade of Ca^+2^ channels [51]. The Ca^+2^ channel blocking activity of Ir.Cr was further confirmed by the rightward shift of calcium concentration response curves in isolated rabbit jejunum preparation in a manner similar to verapamil. Calcium channel blockers are an essential class of drugs demonstrating dose-dependent inhibition of Ca^+2^ influxes [52].

The Ir.Cr was found to cause relaxation of both carbachol (1 μM)- and K^+^(80 mM)- induced contractions in isolated rabbit tracheal preparations and such non-specific relaxant effect is likely to be mediated through Ca^+2^ channel blockade [53] .

Moreover, Ir.Cr exerted relaxant effect on application to isolated rabbit aortic preparations and also relaxed phenylephrine- and K^+^ (80 mM)-induced contractions. The isolated rabbit aortic preparation has been used to elaborate mechanism of calcium channel blocking activity [25,26] as K^+^ (80 mM)-induced contractions are mediated through activation of Ca^+2^ channels as well as release of Ca^+2^ from endoplasmic reticulum, whereas mechanism underlying the phenylephrine-induced contractions is through the activation of α-adrenergic receptors and subsequent Ca^+2^ influx through the receptor mediated Ca^+2^ channels. The Ir.Cr was able to relax both phenylephrine- and K^+^ (80 mM)-induced contractions likely to mediate through Ca^+2^ channel blockade. The presence of alkaloids and saponins as the plant constituents, may explain the gut stimulant actions of the plant extract as these are believed to possess gut stimulatory properties.

Antiemetic activity was performed at doses (50 mg/kg, 100 mg/kg, 150 mg/kg, 200 mg/kg). 150 mg/kg was observed to be more potent antiemetic dose. Analgesic activity was performed at doses (100 mg/kg, 200 mg/kg, 300 mg/kg). 200 mg/kg showed effective analgesia. Antipyretic activity was performed at doses (50 mg/kg, 80 mg/kg, 10 mg/kg). 80 mg/kg of the crude extract was potent antipyretic. In these activities dose higher than the potent dose was found to be toxic. Antioxidant activity was performed *in vitro*. It was not tested in vivo.

The antioxidant potential of Ir.Cr was explored through *in vitro* studies. The free radical formation and reactive oxygen and nitrogen species are involved in various ailments including cancer, arthritis, heart diseases, immune defects and neurodegenerative disorders including aging process. Hence, use of Ir.Cr may play a role in amelioration of disease process of above mentioned diseases due to itsantioxidant activity.

Moreover, Ir.Cr was found to be a good inhibitor of acetylcholinestrase and butyrylcholinesterase and both enzymes play a significant role in modulation of activity level through increase in acetylcholine levels at synaptic clefts. Several agents capable to inhibit acetycholinesterase are valuable for the management of disease conditions like *myasthenia gravis*, characterized by increased muscle weakness and intense fatigue [54-56]. Similarly, acetycholinesterase inhibitors have also been used in Alzheimer’s disease, in which the cholinergic impairment caused dementia and other nervous problems [57]. Few other plants have been reported to share this capability to inhibit acetylcholinesterase and have shown therapeutic potential against the Myasthenia gravis and Alzheimer’s disease, e.g., *Salvia lavandulaefolia*[58,59] and *Salvia chionthana*[60].

Furthermore, Ir.Cr caused significant inhibition of lipoxygenase enzyme, which is known to cause conversion of arachidonic acid into leukotrienes (LTs) [61], whereas LTs C4, D4, and E4, collectively known as cysteinyl LTs, are products of 5-lipoxygenase [62]. Initially, these were reputed as potent constrictors of respiratory tract but it has been subsequently realized to cause inflammation, increase in capillary permeability and increase in mucus secretion, which may exacerbate asthma and allergic rhinitis. These are known to be mediated through binding of cysteinyl LTs to the cysLT receptor 1 (CysLT1), hence, antagonism of CysLT1 and inhibition of 5-LO are reported to have therapeutic potential to manage asthmatic condition [63]. We can hypothesize that the inhibition of lipoxygenase by Ir.Cr may be useful in management of asthma and allergic rhinitis.

The Ir.Cr was found to exhibit antipyretic activity as it caused inhibition of pyrogen-induced pyrexia. The pyrexia is caused by the access of pro-inflammatory mediators (prostaglandins and other metabolites of arachidonic acid) to thermostat in hypothalamus; hence pyrexia is an outcome of disturbed thermostat in hypothalamus [64]. It is possible that the observed antipyretic effect is mediated by a limited availability of prostaglandins through inhibition of cyclooxygenase, as it has already been found to inhibit lipoxygenase.

The pain sensation is generated by interaction of prostaglandins with pain receptors [65,66]. The prostaglandins are produced by action of cyclooxygenase 1 and cyclooxygenase 2 on ω-3 and ω-6 C20 fatty acids [67]. The methanol extract of *Isodon rugosus* demonstrated a significant analgesic effect in tail flick experiments performed on mice, and this is likely mediated through theinhibition of cyclooxygenase, resulting in a limited availability of prostaglandin for action on nociceptors. It also indicates central mediated nociception through opioid receptors.

The Ir.Cr demonstrated antiemetic properties *in-vivo* in chicks after administration of copper sulphate. The vomiting centre lies in the *medulla oblongata*, by activation of motor pathways descending from this centre. The vomiting centre can be activated directly by irritants or indirectly following input from 4 principal areas, i.e., gastrointestinal tract, cerebral cortex and thalamus, vestibular region, and chemoreceptor trigger zone (CTZ). The CTZ is in vicinity to medulla and contrary to other brain centres it is not protected by the blood-brain barrier [68]. The observed anti-emetic effect of Ir.Cr can be likely mediated through inhibition of CRTZ.

## Conclusions

The observed relaxant effect on isolated rabbit jejunum, trachea and aorta preparations showed by the methanol extract of *Isodon rugosus* can be likely mediated through Ca^+2^ channel blockade and may provided scientific basis to validate the folkloric uses of the plant in the management of gastrointestinal, respiratory and cardiovascular ailments. The observed antioxidant activity as well as the lipoxygenase inhibitory activity of Ir.Cr may validate its folkloric use in pain and inflammations. We used crude extract of plant which is a combination of multiple constituents. So exact constituent responsible for these activities should be pinpointed by conducting further research and exploring the individual constituent. The bioactive constituent responsible should be isolated, quantified and its structure should be elaborated by analytical techniques.

## Competing interests

The authors declare that they have no competing interests.

## Authors’ contributions

KHJ, JA, FS and MA designed and carried out the experimental work. II and MZUH analyzed the statistical data and interpretation of results. HZEJ and VDF drafted and critically evaluated the manuscript. All authors read and approved the final manuscript.

## Pre-publication history

The pre-publication history for this paper can be accessed here:

http://www.biomedcentral.com/1472-6882/14/71/prepub
